# Transient knockdown-mediated deficiency in plectin alters hepatocellular motility in association with activated FAK and Rac1-GTPase

**DOI:** 10.1186/s12935-015-0177-1

**Published:** 2015-03-07

**Authors:** Chiung-Chi Cheng, Yen-Chang Clark Lai, Yih-Shyong Lai, Yung-Hsiang Hsu, Wei-Ting Chao, Kee-Chin Sia, Yu-Hui Tseng, Yi-Hsiang Liu

**Affiliations:** Department of Pathology, Chang Bing Show Chwan Memorial Hospital, No. 6, Lugong Rd., Lugang Town, Changhua County 505 Taiwan; Center for General Education, Providence University, Taichung City, Taiwan; Department of Pathology, Kaohsiung Medical University Hospital, Kaohsiung City, Taiwan; Department of Pathology, Tzu Chi University, Hualien County, Taiwan; Department of Life Science, Tunghai University, Taichung City, Taiwan

**Keywords:** Cell motility, Cytoskeleton, Focal adhesion kinase, Hepatocellular carcinoma, Plectin

## Abstract

**Background:**

Plectin is one of the cytolinker proteins that play a crucial role in maintaining the integrity of cellular architecture. It is a component of desmosome complexes connecting cytoskeletal proteins and trans-membrane molecules. In epithelial cells, plectin connects cytokeratins and integrin α6β4 in hemidesmosomes anchoring to the extracellular matrix. In addition to the function of molecular adherent, plectin has been reported to exhibit functions affecting cellular signals and responsive activities mediated by stress, cellular migration, polarization as well as the dynamic movement of actin filaments. Plectin deficiency in hepatocellular carcinoma results in abnormal expression of cytokeratin 18 and disassembled hemidesmosome. Therefore, it is hypothesized that the plectin deficiency-mediated collapse of cytoskeleton may modulate cellular motility that is associated with consequent metastatic behaviors of cancer cells.

**Methods and results:**

The cellular motility of plectin-deficient Chang liver cells generated by transient knockdown were analyzed by trans-well migration assay and the results revealed a higher migration rate. The confocal microscopy also demonstrated less organized and more polarized morphology as well as more focal adhesion kinase activity in comparison with that of the mock Chang liver cells. Furthermore, plectin-knockdown in Chang liver cells was associated with a higher activity of Rac1-GTPase in accordance with the results of the Rac1 pull-down assay. The immunohistochemical assay on human hepatocellular carcinoma showed that the expression of focal adhesion kinase was increased in the invasive front of tumor.

**Conclusion:**

Plectin-deficient human hepatic cells exhibit higher cell motility associated with increase in focal adhesion kinase activity that are comparable to the properties of invasive hepatocellular carcinoma.

## Background

The cytoskeletal protein networks including microtubules (MTs), microfilaments (MFs), and intermediate filaments (IFs) are essential to maintain the integrity of eukaryotic cells. Proper cross-linking structures among these cytoskeletal proteins are crucial for intracellular architectures and normal cellular morphology. Plectin is a versatile adherent macromolecule expressed in a wide range of mammalian cells with a molecular weight of 500 kDa [1]. Previous studies revealed that plectin resembles with vimentin filaments in the processes of focal adhesions (FAs) and mediates the polymerization of fibronectin fibrils while fibrillar adhesions occur. The macromolecular assemblies result in a cage-like core structure maintaining a stable nucleus position while the cells are associating with extracellular matrix [2]. In addition, plectin is a RACK1 (receptor activated C kinase 1) scaffolding protein affecting protein kinase C (PKC) activities [3], Rho/Rac/cdc42 signaling pathway and actin filaments dynamics [4]. Plectin also participates in regulating mitogen-activated protein (MAP) kinase cascades and the PKC signaling pathway leading to Erk1/2 activation and cell migration [5].

Hemidesmosome (HD) plays a role in anchoring keratinocytes to extracellular matrix. The HD protein complex contains integrin α6β4 binding with the plectin-mediated IFs (cytokeratin). The plectin-binding sites of integrin α6β4 are the second fibronectin type III (FnIII) domain in the β4 subunit and the actin-binding domain of the calponin homologous region [6-8]. It was reported that plectin binds with integrin β4 subunit through its plakin domain [9]. In the processes of wound healing, cellular differentiation and carcinoma invasion, keratinocytes migration is mediated by dynamic assembly and disassembly of HDs. In presence of calcium mediation, calmoldulin modulates the binding between integrin α6β4 and plectin isoform 1a in the differentiating keratinocytes [10].

Microenvironment changes in mechanical properties have been found in the tissues surrounding neoplasms. In particular, the focal adhesion kinase (FAK) is involved in regulating many biomechanical processes such as cell cycle progression, apoptosis and cell migration [11]. FAK is a cytoplasmic tyrosine kinase resembling with focal adhesions and consequently transduces intracellular signals regulating cell adhesion, actin-myosin dynamics, cell motility and angiogenesis that are perturbed in cancer cells [12]. The increased expression of FAK has been found in several types of human cancer [13,14].

Parenchymal cells count up to 80% of human hepatocytes. Two types of cytokeratins (CKs), CK8 (type II) and CK18 (type I) with molecular weight of 52kDa and 45kDa respectively, are expressed and compose of the major components of IFs in human hepatic parenchyma cells [15]. Our previous studies demonstrated that plectin-deficiency-mediated pleomorphism is associated with an altered level of CK18 expression in human hepatocellular carcinoma (HCC) [16,17]. Given the fact of that plectin is essential for binding the trans-membrane integrin α6β4, the impact of plectin-deficiency on the assembly between the intracellular IFs network and extracellular matrix is interested to be elucidated. In the present study, transient plectin-knockdown in Chang liver cells was analyzed for cell migration and the Rac1-GTPase activity. The cellular morphology was also observed. Furthermore, HCC specimens were collected for investigating the levels of plectin and FAK by immunohistochemical methods.

## Results

### Plectin-knockdown Chang liver cells showed a higher rate of cell migration

The results of trans-well migration assay demonstrated that plectin-deficiency in Chang liver cells derived from transient knockdown revealed a significant higher rate of cell migration (about 300%, *p < 0.001*) compared with that of the mock counterpart (Figure 1).

**Figure 1:** **Plectin depletion enhanced Chang liver cell migration.** Plectin siRNA-transfected Chang liver cells were transferred to trans-well migration insert, followed by 4 hour incubation as described in the section of “materials and methods”. Plectin-knockdown Chang liver cell (refer to as Plectin siRNA) significantly showed a higher level of cell migration. Data are presented as mean ± standard error obtained from three independent experiments, *** indicates p < 0.001. The migrated cell number of mock group was assumed as 100%. Cell migration of plectin-knockdown Chang liver cell is presented as the ratio to that of the mock group.

### Rac1-GTPase activity was higher in plectin knockdown Chang liver cell

In Figure 2, the results of Western blotting assay showed an increase in Rac1-GTPase activity in the lysate of siRNA-transfected cells, suggesting that the depletion of plectin in hepatic cells might be associated with the activation of Rac1-GTPase activity. The dramatic decrease in the amount of plectin (top panel of Figure 2a) demonstrated effective knockdown of plectin gene by adding siRNA.

**Figure 2:** **Plectin-knockdown Chang liver cells appears to have increased Rac1-GTPase activity.** Total lysate separately prepared from mock cells and plectin siRNA-transfected cells were applied to Rac1-GTPase pull-down assay and Western blotting assay with anti-Rac1 and anti-plectin antibodies. **(a)** The result showed that the Rac1-GTPase level was increased in plectin-knockdown cells. **(b)** The results indicated the quantification of Rac1-GTPase level. Values are presented as mean ± standard error obtained from three independent experiments, * indicates p < 0.05.

### FAK activation and cellular morphology changes were associated with plectin-deficient hepatic cells

In this study, the results of immunofluorescent microscopy revealed that increased FAK activation along the cellular edge was associated with the plectin-knockdown Chang liver cells (Figure 3). Induction of action stress fibers was also observed in the plectin-deficient cells. In addition, the plectin-knockdown Chang liver cells were amorphous under more polarized microscopy. These results suggested that plectin deficiency in hepatic cells is associated with morphological transformation and dynamic focal adhesion that are the phenomenon of invasiveness.

**Figure 3:** **Plectin-knockdown Chang liver cells possess distinct cell morphology and FAK activity.** Plectin siRNA-transfected Chang liver cells were fixed and stained with anti-plectin and anti-FAK antibodies. Confocal micrographs demonstrated that plectin-knockdown Chang liver cells were polarized and with less regularity in cellular arrangement. More induced actin stress fibers (arrowheads) and higher FAK activity (arrows) were shown at the cell edges. Scale bar = 10 um.

### The expression of plectin in human HCC tissues

The expression of plectin in HCC tissues showed different expression patterns of plectin from that of the non-tumor tissues. As shown in Figure 4a, the pleomorphic tumor cells were arranged in irregular nests and plectin-staining revealed weak signals. In contrast, the hepatocytes appeared uniform cuboid arranged in sheets or plate pattern with strong plectin signals in the non-tumor cytoplasm. It implied that decreased plectin expression is accompanied with human hepatic carcinoma.

**Figure 4:** **Expression of plectin and FAK phosphorylation in hepatocellular carcinoma. (a)** Immunohistochemical analyses on the paraffin-embedded samples of human hepatocellular carcinomas and non-tumor liver tissues were detected by the use of anti-plectin antibody (×200). Plectin was detected with stronger signals in non-tumor liver tissue (lower left area) whereas HCC tissues showed weak signals (upper right area). **(b)** The results of immunohistochemical analysis on paraffin-embedded samples of HCC tissues by using anti-FAK antibody. The expression FAK was higher at the invasive front of tumor. In contrast, the central part of tumor revealed lower FAK expression with weak signals.

### The expression of FAK in the invasive tissues of human HCC

In the trans-well migration assay, plectin-knockdown Chang liver cells had a higher rate of cell migration. Increased activities of Rac1-GTPase and FAK were also demonstrated. Furthermore, human HCC with higher levels of FAK activation in the invasive tissues were also detected *in situ*. In Figure 4b, higher activation of FAK was found at the invasive front of HCC compared to the non-invasive part around the center of tumors. The *in situ* immunohistochemical data suggests a possible correlation between the higher FAK activation and the invasiveness of cancer cells with plectin deficiency.

## Discussion

Along with microtubules and actin filaments, intermediate filaments are major components of the cytoskeleton in metazoan cells and play a role in providing stable cellular morphology under different conditions. Our previous studies have elucidated that the involvement of plectin in regulating the cytoskeletal organization in human liver cells. Plectin-deficient hepatocytes revealed alteration in the expression and the organization of CK18. In consequence, partially augmented cytoskeletons were associated with pleomorphic changes that were comparable to the properties of human HCC [16,17].

Metastasis is a major factor leading to cancer-related mortality [18]. Identification of the risk factors associated with cancer metastasis is an important issue for improving clinical management. For every single cell, migration is fundamental activity involving the processes of differentiation, wound healing, and cancer metastasis. While cellular migration occurs, coordinated cytoskeleton, anchoring proteins and cytolinker proteins are essential for proper movement [19]. Therefore, understanding the mechanisms of cellular migration will be helpful to develop strategies alleviating cancer metastasis.

In keratinocyte, plectin isoform 1a requires calmodulin to modulate integrin α6β4 during the cellular differentiation mediated by calcium ions [10]. Plectin is the molecule anchoring IF to HDs by connecting the β4 FnIII domains of integrin with its actin binding region and plakin domain. When the concentration of calcium ion is increased, Ca-camodulin complex interacts with the actin binding domain of plectin and dissociates plectin from integrin. Up to the present, the role of actin filament-integrin assembly on cellular motility remains unclear. Hehlgans and colleagues [20] reported that a conformational change of integrin mediated by its association with extracellular matrix gives rise to clustered integrin. The aggregated trans-membrane proteins activate signaling cascades that in subsequence mediate the formation of focal adhesion complexes. The dynamic assembly between actin-filaments and integrin triggers cellular movement and creates cellular adhesion to substratum sites. Focal adhesions play essential role in cell motility in a growing tissue culture [21,22]. In this study, the plectin-knockdown human liver cells revealed higher level of cell motility by enhancing the FAK activity. In accordance, we propose a hypothesis that the association between integrin and actin may be mediated by active FAK modulated by plectin-Ca-camodulin complex. In human HCC, deficiency in plectin may create more free integrin FnIII domains adapting for active FAK that is required for macromolecular assembly prior to tumor cell migration. In future, it deserves more efforts to investigate the molecular mechanism involved in plectin deficiency-mediated changes in cell morphology and motility.

Plectin, a member of plakin family, plays several pivotal roles to maintain cellular architecture by connecting cytoskeleton and/or by modulating activity of kinases. In the filamentous structure of HD, plectin connects CK18 and integrin α6β4 and the complex affects cell motility. Rac1 exhibiting GTPase activity belongs to the Rho family. The Rac1-GTPase with small molecular weight (21 kDa) modulates several important cellular processes including migration, adhesion and differentiation by regulating cytoskeletal relocation and activation of protein kinases [23]. In the front edge of the migrating cells, activated Rho GTPase is associated with actin polymerization leading to the formation of lamellipodia. A branched structure in lamellipodia where actin filaments assembly occurs consists of the Rac1-GTPase activated WAVE protein and Arp2/3 complex [24]. The higher Rac1-GTPase activity indicates the higher level of cell motility. The results in this study indicated that enhanced cell motility in plectin-knockdown Chang liver cells was associated with increased Rac1-GTPase activity and cell migration. In terms of cell morphology, the plectin-knockdown Chang liver cell became more polarized and showed a less degree of regularity of cell arrangement. Regarding to the distribution of active FAK, the cell edges of plectin-deficient Chang liver cells were comparable to the invasive front of HCC tissues.

## Conclusions

All the previous results discussed in this report support our hypothesis that plectin may be correlated with the regulation of cell motility involved in the invasiveness of hepatic carcinoma. This study also provided related mechanisms associated with the activation of FAK and Rac1-GTPase.

## Methods

### Antibodies

Mouse anti-Rac1 monoclonal antibody was purchased from Thermo Scientific. Goat anti-plectin antibody was purchased from Santa Cruz Biotechnology (Santa Cruz, CA, USA). Mouse anti-phosphorylated FAK monoclonal antibody (anti-FAKp) was acquired from BD Transduction Laboratories™ (Franklin Lakes, New Jersey, USA). Secondary antibodies including Cy2-conjugated anti-mouse IgG and Cy3-conjugated anti-goat IgG used for immunofluorescence microscopy, horseradish peroxidase-conjugated goat and mouse antibodies used for Western blotting analysis, as well as biotin-conjugated goat and mouse antibodies used for immunohistochemistry were purchased from Jackson Immuno Research Laboratories (West Grove, PA, USA).

### Cell cultures

Chang liver cells (CCL-13, obtained from ATCC) were derived from normal human hepatic tissue. Dulbecco’s minimum essential medium (DMEM) supplemented with 10% fetal bovine serum, 50 unit/ml penicillin and streptomycin was used for culture at 37°C in presence of 5% CO_2_. Medium was replaced and confluent growth was split regularly.

### HCC tissue specimens

Five primary HCC specimens without prior neo-adjuvant therapy were obtained from surgical resection operated in the Department of Surgery, Chang Bing Show Chwan Memorial Hospital, Changhua County, Taiwan. Pathological diagnosis confirmed that all specimens were neoplastic grade II. Paraffin-embedded blocks of the specimens were prepared as usual protocols.

### Transient knockdown of plectin in Chang liver cells

To study the biological effects of plectin deficiency, transient knockdown was performed by using RNA interference techniques. Small interfering RNA (siRNA) specific for plectin transcripts was purchased from Dharmacon, Inc. (Lafayette,CO). The pre-designed siRNA kit contains a mixture composed of four fragments of siRNA targeting to the sequences of conserved regions encoding all plectin isoforms. Chang liver cells were grown on a 60mm petri dish to 60% confluence. For introducing the siRNA into cells, the siRNA was diluted with serum free medium (1:100, v/v) and then gently mixed with pre-diluted (1:50, v/v) Lipofectamine 2000 (Invitrogen, USA). The mixture was left at room temperature for 20 minutes. Afterwards the mixture was added to the petri dishes with gentle shaking. The transfected culture will be available for further assays after 48 hours.

### Trans-well migration assay

Cell motility was examined by using QCM™ 24-Well Colorimetric Cell Migration Assay kit (Millipore). The siRNA-transfected Chang liver cells were harvested and then transferred into the 24-well plate inserted with trans-well. Cellular migration was determined in accordance with the manufacture’s protocol.

### Preparation of p21-activated kinase (Pak)

The Pak-expressing E.coli BL21 strain was grown in 500ml ampicillin supplemented-LB medium to the density with OD_600_ value 0.6-0.8. Pak expression was induced by adding 500μL isopropyl β-D-1-thiogalactopyranoside (1mM) and maintains further shaking at 4°C for 3 hours. The bacterial culture was harvested by centrifugation (6000g) at 4°C for 15 minutes and the pellet was washed with 25ml washing buffer containing 62.5μL phenylmethylsulfonylfluoride (PMSF), and 250μL protease inhibitors cocktail. The washed bacteria were lysed by sonication (Misonixsonicator 3000) as protocol’s instruction. The lysate was added with 500μl Triton X-100 and incubated at 4°C for 30 minutes. The supernatant was collected after centrifugation (12000g) at 4°C for 20 minutes. The glutathione S-transferase (GST)-conjugated beads (200μl) was added to the collected solution and incubated at 4°C for 30 minutes with continuous shaking. The Pak-bound beads were further collected by centrifugation (5000rpm) at 4°C for 3 minutes and then washed with 1ml 1x phosphate buffered saline (PBS) buffer. The washing procedures were repeated for 3 times. The Pak-GST-conjugated beads can be collected and suspended with 1ml lysis buffer (25mM Tris-base, 150mM NaCl, 1% NP-40, 5% Glycerol, 1mM ethylenediaminetetraacetic acid (EDTA), 100μM sodium orthovanadate, 200μM PMSF and protease inhibitors cocktail).

### Ras-related C3 botulinum toxin substrate 1 (Rac1)-GTPase pull-down and detection assay

A 60mm petri dish culture of mock and plectin knockdown Chang liver cell were separately harvested and suspended with lysis buffer (25mM Tris-base, 150mM NaCl, 1% NP-40, 5% Glycerol, 1mM ethylenediaminetetraacetic acid (EDTA), 100μM sodium orthovanadate, 200μM PMSF and protease inhibitors cocktail). Supernatant of both samples were collected by centrifugation (11000g) at 4°C for 10 minutes. The protein concentrations were determined by bicinchoninic acid assay (BCA assay) and adjusted to a final amount of 500μg in a volume of 700μl. The Pak-GST-conjugated beads (10μl) prepared as the previous description was then added to each samples and were continuously shaken at 4°C for 2 hours. The incubated samples were further washed with lysis buffer and collected by centrifugation (4500rpm) at 4°C for 5 minutes. The washing procedures were repeated for three times. The washed samples were rinsed with distilled water and were eligible for determining the Rac1-GTPase activity by Western blotting analysis.

### Western blotting analysis

Total cellular lysate and Rac1-GTPase pull-down complex were separately loaded for running a 10% sodium dodecyl sulfate polyacrylamide gel (SDS-PAGE). Followed by the completion of electrophoresis, the gel was transferred onto a polyvinylidene difluoride (PVDF) membrane by using semi-dry transferring method (Bio-Rad). The transferred membrane was blocked with 5% non-fat milk (in phosphate buffered saline with Tween-20 (PBST) buffer) for 1 hour and then washed three times for 5 minutes with PBST prior to adding the diluted primary antibody (1:1000 in PBST). The hybridization was undergone for one hour and the hybridized membrane was washed with PBST three times for 5 minutes prior to adding the diluted secondary antibody (1:5000 in PBST). At last, the chemiluminescent reagent was added to the washed membrane and the image was developed by the Chemiluminescence Imaging System (Fuji, Japan) as manual’s instruction.

### Immunofluorescent assay

The plectin siRNA-transfected Chang liver cells were grown in a 24-well plate (4 × 10^3^ cells per well) for 48 hours. Cells were washed with ice-cooled PBS (137mM NaCl, 2.7mM KCl, 8mM Na_2_HPO_4_ and 1.5mM KH_2_PO_4_, pH7.4) and fixed with 3.7% paraformaldehyde at room temperature for 20 minutes. The fixed cells were washed with PBS for three times and then treated with 0.1% Triton X-100 for 2 minutes. After three times washing with PBS, mouse anti-FAKp (1:100 in PBS) and rabbit anti-plectin (1:100 in PBS) antibody were simultaneously added to the pre-treated cells for 1 hour. For fluorescent imaging, cells were incubated with secondary antibodies (Cy2-conjugated anti-mouse IgG and Cy3-conjugated anti-goat IgG) and Cy5- conjugated Phalloidin dye (1:100 in PBS) for 1 hour. After three-time washing with PBS, fluorescent images were viewed under the Zeiss LSM 510 confocal microscope.

### Immunohistochemistry analysis

The paraffin-removed sample sections were rehydrated and treated with 3% H_2_O_2_ for 10 minutes to eliminate the endogenous peroxidase activity. Non-specific binding were blocked with bovine serum albumin for 10 minutes. The sample sections were incubated with anti-plectin (1:40 dilution) and anti-FAKp (1:50 dilution) monoclonal antibodies for 1 hour at room temperature. The biotinylated anti-goat and anti-mouse IgGs were then added (1:400 dilution) and incubated at room temperature for 1 hour. The specific bindings were detected by adding avidin-conjugated peroxidase and observed under a light microscope (BX51; Olympus, Tokyo, Japan) in presence of the substrate reagents. For each HCC specimen, the immunohistochemistry assay was triplicated on separate sample sections.

## Abbreviations

CK18: Cytokeratin 18
CKs: Cytokeratins
FAK: Focal adhesion kinase
FAs: Focal adhesions
FnIII: Fibronectin type III
GST: Glutathione S-transferase
HCC: Hepatocellular carcinoma
HD: Hemidesmosome
IFs: Intermediate filaments
MAP: Mitogen-activated protein
MFs: Microfilaments
MTs: Microtubules
Pak: p21-activated kinase
PBS: Phosphate buffered saline
PBST: Phosphate buffered saline with Tween-20
PKC: Protein kinase C
PMSF: Phenylmethylsulfonylfluoride
Rac1: Ras-related C3 botulinum toxin substrate 1
RACK1: Receptor activated C kinase 1
siRNA: Small interfering RNA
